RETRACTED

# Does green investment affect environment pollution: Evidence from asymmetric ARDL approach?

**DOI:** 10.1371/journal.pone.0292260

**Published:** 2024-04-18

**Authors:** Yanan Shen, Saif Ur Rahman, Nabila Shahzadi Hafiza, Muhammad Saeed Meo, Muhammad Sibt E. Ali

**Affiliations:** 1 School of International Business, Southwestern University of Financial and Economics, Chengdu, China; 2 Faculty of Economics and Commerce, The Superior University, Lahore, Punjab, Pakistan; 3 Assistant Professor in Finance, Department of Economics & Finance, Sunway University Malaysia, Petaling Jaya, Selangor, Malaysia; 4 School of Business, Zhengzhou University Henan, Zhengzhou, China; University of Economics Ho Chi Minh City, VIET NAM

## Abstract

Pollution in the environment is today the biggest issue facing the globe and the main factor in the development of many fatal diseases. The main objective of the study to investigate green investments, economic growth and financial development on environmental pollution in the G-7 countries. This study used annual penal data from 1997 to 2021. The panel NARDL (Non-linear autoregressive distributed lag) results affirm that the positive change of green investment and negative shock in green investment have a significant and positive association with environment pollution in G-7 nations. Our findings provide more evidence for the long-term asymmetry between financial development and environmental performance. However, the findings confirm that a positive modification in financial development has a positive and significant effect on environment pollution. Whereas negative shock in financial development is negative and insignificant relationship with environment pollution. Moreover, the outcomes of the study reveal that both positive shock in gross domestic product growth and negative shock of economic growth have a significant and positive link with environment pollution in G-7 countries. According to the findings, by lowering carbon dioxide emissions, green investments reduced environmental pollution in the G-7 nations over the long and short term. Moreover, it is an innovative research effort that provides light on the connection between green investments, financial development, and the environment while making mention to the EKC in G-7 countries. After all these, our recommendation is to increases green investment expenditures to reduce environmental pollution in the G-7 nations based on our findings. Additionally, one important way for the nation to achieve its sustainable development goals is to improve advancements in the financial sector.

## Introduction

Significant global changes have been experienced over the past 65 years, including global warming and the observed and expected climate changes for the twenty-first century. The impact of climate change (CC) on many aspects of the ecological, environmental, sociopolitical, and socioeconomic disciplines makes it an intergovernmental complicated challenge on a worldwide scale [1]. The greatest problem abutting the world currently is environmental degradation, which is also the primary cause of numerous deadly diseases. Emerging nations like the G-7 share this concerning recent domestic and international policy talks have increasingly focused on climate change and environmental degradation. An indicator of environmental pollution, CO2 emissions have been rising quickly around the globe. From 33.1 Gt CO2, global carbon emissions grew by 1.7% in 2019. Lung conditions and other potentially fatal diseases are frequently brought by environmental pollution. Environmental contamination has consequently developed into a significant issue [2]. Accelerating as a result of rapid exploration, mining, and industrialization. Despite widespread awareness, environmental contamination continues to cause human suffering. The three primary forms of environmental pollution that have an impact on the entire globe are contamination of the air, water, and soil [3]. Pollution is bad for us. In addition, even if greenhouse gas emissions are decreased, their effects will still be felt. As a result, agreements like the Paris Accords in 2016 demand that all countries lower their emission levels to some extent while also taking into consideration laws and regulations that help in human adaptation to climate change [4].

RETRACTED

Additionally, Iceland is a country that has made a bold promise to significantly cut GHG emissions in the following five important industries by 2030: Energy production and small industry (to reduce greenhouse gas emissions by 67%), waste management (to reduce greenhouse gas emissions by 66%), ships and ports (to reduce greenhouse gas emissions by 42%), land transportation (to reduce greenhouse gas emissions by 21%), and agriculture (to reduce greenhouse gas emissions by 5%) are the targets for 2020, according to the Ministry for the Environment and Natural Resources. With this initiative, Iceland is on track to meet its goal of becoming carbon neutral by 2040 by reducing GHG emissions by around 40% by the deadline, particularly in the ESR sectors. This dedication is seen in the country’s updated Climate Action Plan (CAP) 2020, which outlines the 48 initiatives the government is now pursuing. It is obvious that the nation’s CAP 2020, which takes into account the Sustainable Development Goals of the United Nations, has a major prediction of lowering GHG emission in the ESR-sectors [4]. Furthermore [5], mentioned that sustainable development goals (SDGs) seek to enhance the quality of the planet’s environment by supplying affordable, dependable, and modern energy sources, which may help lessen the negative environmental effects of economic activity for a higher standard of living (SDGs, 2021).

RETRACTED

The comprehensive long-term patterns in temperature and precipitation, as well as other factors like atmospheric pressure and humidity, are used to define climate change. In addition, some of the most well-known domestic and international repercussions of climate change include the unpredictable weather patterns, melting ice sheets around the world, and the consequent heightened sea level rise [1].

Emissions of carbon dioxide (CO2) around the world have risen rapidly. Global carbon emissions reached 36 billion tons in 2020, an increase from 1.6 billion tons in 1990. The steady reliance on dirty energy sources, which is bad for the environment, could be to blame for the rise in emissions. Between 1970 and 2020, global CO2 emissions increased by approximately 91%, with fossil fuel combustion and industrial operations accounting for 79% of total CO_2_ emissions, according to the Environmental Protection Agency (EPA). As a result, global emission-mitigation policies must be implemented due to the alarming rate of increase in CO_2_ emissions [6–8].

Some studies in the environmental economics literature have addressed investment issues, particularly green investment, in light of the significance of reducing traditional energy consumption and combating the growing problem of pollution. Economic expansion, low interest rates, high fuel prices, and environmental regulation all appear to encourage green investment, according to previous studies [4, 9, 10]. Liao and Shi discovered that by increasing the severity of environmental regulations, public appeal can encourage green investment by businesses. The available literature is scant when it comes to the function that green investments play. Financial support for addressing climate challenges is provided by green investment policy based on the debt capital market [11]. It affects the pattern of private capital mobilization for clean energy development and makes low-pollution projects more cost-competitive [12]. Effective energy systems and climate markets are the result of green investment, which significantly reduce pollution emissions and promote sustainable development [12, 13]. Increased capital investment in green technology can reduce the negative impact of enterprise production activities on the environment by enhancing enterprises’ production efficacy and realizing the replacement of nonrenewable energy with renewable energy [10, 14]. According to [15] who looked into the effects of the Czech Republic’s green investment plan, the federal subsidy policy for biomass boilers and heat pumps cut greenhouse gas emissions. Sachs and others Green bonds and green funds are important tools for achieving the Sustainable Development Goals (SDGs) and low-carbon development, according to a study conducted in 2019 that attempted to evaluate the impact of green investment and projects on the SDGs. However [16], discovered that while green investment has a positive effect on the consumption of clean energy in the short term, it has little effect on carbon emissions in the long run

Green investments may minimize environmental pollution in a variety of ways, including the efficiency of energy saving and emission reduction, the growth of technical innovation capabilities, and the modernization of the industrial structure. The environmental crisis that has developed as a direct result of a variety of forms of pollution, the rapid exploitation and use of natural resources, a growing reliance on energy-intensive and ecologically damaging technology, excessive use of hazardous pesticides and herbicides, the eradication of invasive species, the loss of a variety of plants due to agriculture and climate change [17]. Deforestation and forest destruction result in emissions that must be reduced through green investments. Even though it is difficult to address this environmental issue using economic tools like taxes, fines, and charges, it is possible to reduce deforestation and climate change with competent governance [18]. According to [19], reducing carbon dioxide emissions requires technological advancement. In developing nations, the demand for energy has increased as a result of the rising use of ICT products. Its significant Environmental contamination may be impacted by carbon dioxide emissions [20, 21].

RETRACTED

As a specific threshold is crossed, the quality of the environment starts to improve. Initially, it declines during growing. The environmental Kuznets curve (EKC), often known as the inverted U-shaped GDP-pollution pattern [22]. Between 1991 and 1995 [41], discovered it for the first time. The scale impact of investor receptivity to green investments and increased electricity demand are frequently cited as the causes of the early negative impacts of economic development on air durability. Yet, the method and/or component influence would ultimately have a positive influence on the environment [23, 24]. When expansion is prioritized over environmental quality in the early phases of development, there are more economic activities (transportation, industrial output, and deforestation) and energy usage. Environmental pollution degrades as a result [23, 24] and the composing impact would be advantageous for the environment in the long term. In the initial stages of growth, there are more economic activities (transportation, industrial output, and deforestation) and energy consumption since expansion is valued more highly than air sustainability. As a result, the environment is becoming less healthy. People inside the second phase of growth seek a cleaner environment in order to reach a higher quality of life as income levels rise as a consequence of the technology effect [22, 25]. Furthermore, If the technical effect takes precedence over the size effect and the component effect, then green investment transparency helps to enhance environmental pollution [22]. When environmental protection is stronger than the capital-labor effect, green financial accessibility can also improve environmental quality through equity channels [26].

The majority of research used carbon dioxide (CO_2_) as one of the environmental quality measures [27–29]. A substantial portion of Muslim nations, the region with the least quantity of EKC research, and a collection of fifty-seven economies make up the Organization of Islamic Cooperation (OIC). [30] estimates that the G-7 countries account for 23.8% of global population. The G-7’s manufacturing employment is rising as a result of globalization and its willingness to accept green investments. This increases the use of renewable resources and energy, which in turn increases pollution, according to [31, 32]. Several countries committed to reduce GHG emissions in order to lower global temperatures as part of the Paris Agreement, which was signed in order to solve environmental challenges. 43 of the 166 nations that have approved this pact are G-7 members [30]. In addition, material exhaustion and ecological scarcity might lead to socioeconomic tensions within the G-7 [33, 34]. Examining the relationship between environmental harm and green investment as well as how they affect EKC for G-7 countries is the goal of this study. Despite the fact that many academics have examined the impacts of openness and green investment on the environment in various countries, there is very little comprehensive literature on the subject for the G-7 [32, 35].

There are currently a few studies that evaluate the environmental nexus between green investment and EKC in G-7 nations. As a result, examination contributes towards the current body of knowledge in many different ways that are consistent with the preceding discussion:(i) it is a first study which illuminates the relationship between the green investment, financial development and environment with allusion to EKC in G-7 countries,(ii) In contrast to previous empirical studies, this study employs a novel method known as the "panel nonlinear Autoregressive Distributed lag model (NARDL)," which is capable of addressing a number of methodological issues associated with panel data, such as heterogeneity and cross-sectional dependence (CSD).(iii)Most EKC literature simply takes CO_2_ emissions as a measure of environmental pollution, which is insufficient to account for environmental consequences. On the other side, the panel NARDL technique makes advantage of heterogeneous grades and the presumption that the variables can all be accounted for by a single component. Policymakers risk being misled if carbon dioxide emissions are the only sign of environmental contamination. As a result, more all-encompassing environmental variables are used to produce solid results. As a result, this research considers contemporary environmental issues. Carbon dioxide (CO_2_), (iv) green investment and openness regarding CO_2_ emissions are among the variables that are largely ignored in the existing literature on EKC. In order to prevent specification bias, our models now include openness for green investment, financial development, and economic growth. (v) Governments, and policymakers are interested in studying the G-7 since, while having worse carbon emissions than industrialized nations that are not participants of the G-7, these countries only account for 8.2% of world output and 10.2% of bank financing [30]. vi) Based on the findings, it makes practical suggestions that will open the door to more investigation into the asymmetric relationship between environmental pollution and green investment and its effects on the G-7 countries. This study looks at how economic growth, green investments, and financial development affect in order environmental pollution in the G-7 to test the EKC hypothesis. The new method is called "nonlinear Autoregressive Distributed lag model" (NARDL). When CO_2_ emission is used as an environmental indicator, our findings confirm that all G-7 groups have inverted-U-shaped EKC. However, when CO_2_ is utilized, in both the G-7 as a whole and the G-7 with lower incomes, a U-shaped EKC is seen. The G-7’s policy recommendations on reforming the energy sector, opening up the green investment market, and using bioenergy sustainably should all be upheld.

RETRACTED

The remaining parts of the paper are arranged as follows: The empirical literature on the green investment nexus and EKC is reviewed in the literature review section. The data and methodology section provides an overview. Results and commentary are provided in the results and commentary section. The segment titled Finishing up comments and proposals provides end and strategy suggestions.

### Literature review

The environmental Kuznets Curve and the pollution halo theory are thus examined in this research over the time span of 1990–2020 for 16 European nations. The empirical finding supported the pollution Halo Hypothesis: There is a negative relationship between foreign direct investment and ecological footprints. The inverted U-shaped curve formed by GDP and its square lends credence to the environmental Kuznets Curve theory. Renewable energy had a negative link with ecological footprints, whereas energy structure had a positive correlation. [36] similarly another side [37]. This study uses panel data from 63 emerging and industrialized economies for the years 1990 to 2020 to analyses the relationship between green energy, non-renewable energy, financial development, and economic growth with carbon footprint. The results demonstrate that all variables are co-integrated over the long term. Additionally, the findings show that using non-renewable energy increases carbon footprint while using green energy slows down environmental deterioration and helps to lessen environmental risks. The deterioration of the environment is also significantly impacted negatively by financial development.

The study used a dataset of chosen 13 Asian growing economies from 1995 to 2020 to analyses the dynamic relationship between carbon footprints, nonrenewable energy and renewable energy consumption, financial development and economic growth, and combatting climate change. According to the research, environmental degradation is accelerated by economic expansion and nonrenewable energy use, but over time, consumption of renewable energy reduces the overall negative effects on the environment [38]. This study looks at the effects of technology advancement on the ecological footprints of the G-7 countries between 1990 and 2020. The study used a cross-sectionally enhanced autoregressive distributed lag (CS-ARDL) model. The study’s findings demonstrate how technology progress reduces ecological footprint. Increased use of human capital and renewable energy is also linked to a smaller ecological footprint. Increased GDP development has both short- and long-term effects on the depletion of the natural environment [39].

In a panel of 119 industrialized and developing nations between 2002 and 2018, this study seeks to examine the effects of energy consumption, financial development, and economic development on the ecological footprint. To do this, the study uses the panel unit root and autoregressive distributed lag (ARDL) model. The ARDL results show that the ecological footprint in industrialized countries is positively correlated with a number of characteristics, including energy consumption, financial development, urbanization, globalization, foreign direct investment, and population growth. On the other hand, the ecological footprint in industrialized nations is negatively impacted by the human development index and natural resources [40].

RETRACTED

The current study looks at the possibility of the conventional environmental Kuznets curve (EKC) with an extension for developing industrialized nations like Brazil, China, India, Indonesia, Russia, Mexico, and Turkey (E-7 economies), encompassing the years 1995 to 2019. The study supports the EKC phenomenon’s existence in E-7 economies, where income growth is valued more highly than environmental sustainability. The results of the study show that upgrading of technology lowers pollution levels [39].

[41–44] and many more research on environmental problems have highlighted green investment openness as one of the critical variables that impact environmental quality. In their pioneering study from 1991 [41], investigated the environmental effects of investor receptivity to green projects and discovered a scale impact while controlling for composition and method effects. Moreover, they discovered that a country’s environmental and green investment policies had an impact on the influence of comparative advantage on environmental quality [45]. Using instrumental variables and the gravity framework [27], investigated the consequences of environmental openness to green investments. The openness and policy variables both have negative coefficients. [46] study that looked at the impact of green investment accessibility on environmental quality found that it had a favorable impact on the environment in OECD countries. Similar to this [47], examined the impact of green investment accessibility on the forestry cycle in 142 countries and found that non-OECD countries had an increase in deforestation while OECD countries experienced a slowing in the process. [48] used data from 58 selected nations to evaluate the impact of green investment openness on the environment. Both green investment openness and green investment improved after applying various and simultaneous equations methodologies.

[49] In the G-7, openness to green investments, economic growth, democracy, and environmental quality were examined. Estimates show that growth, democracy, and openness in green investments all had favorable effects on the environment. Additionally [50], this study examines the effects on the environment of the G7 countries’ economic policy uncertainty, economic complexity, renewable energy use, and energy intensity. For a panel dataset from 1997 to 2015, the study uses Fully Modified Ordinary Least Squares and a fixed effect model with resilient standard errors from [51] The results show a long-term association between the relevant variables and ecological footprint and carbon dioxide emissions. Particularly, high energy intensity fuels environmental pollution, while unpredictability in economic policy and the use of renewable energy sources effectively halt environmental deterioration.

RETRACTED

Furthermore, this argument is consistent with [52] assertion that all investments that assist EP ought to be considered GI. Contradictory results have been discovered after extensive research into the connection between GI and EP. The country’s EP improved as a result of investments in clean energy-related research and development projects, according to the findings. On the other hand, investment in nuclear energy projects led to a decline in the country’s EP. From 2000 to 2018, the economies of the E-7, according to [53], benefited from using biomass energy. Furthermore, in China [54], With the help of a novel CSARDL estimator, the study determined that green investments are a positive driver of EP due to their low carbon emissions. [55] looked at major investment economies and found that EP and green investments have a tenuous connection.

The findings indicate that investments in clean energy contributed 11.04 percent of the total change in carbon emissions to global mitigation. [56] demonstrated that gas pollution was reduced by building energy-efficient improvements. From 1980 to 2017 [53], looked at Argentina and found that the best way to improve EP was to invest in renewable energy. [57] took a gander at the US economy and recommended making interests in the land and improvement enterprises to assist with getting carbon non-partisan. Financial development (FD) is defined by [58] as the availability of a wide range of stable, effective, and accessible financial institutions, with a focus on improving economic viability as the main goal. A strong financial system, according to [59] generates local savings that are invested in profitable local businesses, which significantly contributes to economic growth. Innovations in the financial sector also make sound financial strategies easier to implement [60] numerous studies have looked into the relationship between FD and EP. The results, though, are at odds with one another. [61] for instance, looked at the relationships between FD and EP in Turkey from 1965 to 2018. Long-term linkages between the datasets have been found using the RALS cointegration test. Calculations by DOLS show that the country’s FD has a detrimental effect on EP. [62] and many others examined the nonlinear relationship between FD and EP in developing nations in Central Asia and Europe. The findings showed that EP initially declined with continuing FD. The square of FD’s rise in EP across the same time periods provided evidence in favor of the inverted U-shaped idea.

RETRACTED

Resulting to the study, in command to help economies achieve environmental supportability, they would support FD which supports advancements in cleaner production techniques, solar paneling, and electrification as well as low-cost renewable energy sources. More specifically, carbon emissivity’s increased by 0.45–0.79% for every 1% increase in FD. [63] looked at the direct and indirect effects of FD on EP in 88 developing economies between 2000 and 2014. According to system GMM econometric estimates, the five FD indicators increased EP in the corresponding nations. The five FD indicators increased EP in the It was also necessary for there to be a weak financial system in order to test the pollution haven hypothesis (PHH) through FDI and the accessibility of green investment.

The PHH for the two variables came to an end when FD rose above specific thresholds. [64] looked into the contributions that foreign direct investment and economic integration made referring to Venezuela’s move towards a carbon-neutral society. Moreover [65], looked into how FD affected EP in OECD countries. Dynamic panel analysis of data from their study showed that FD increased EP and decreased emissions rates in these economies. It was suggested that investments in FD and energy efficiency be given top priority in order to advance EP.

Considering energy usage and economic growth [66], examined the relationship between FD and EP variables in China. According to the revelations, FD advanced EP all throughout the country. From 1971 to 2018, how FD and EP interacted in Argentina. In 24 different nations between 1970 and 2014 [67], examined the link between FD-EP. The effects of FD on EP are threshold-dependent, as shown by the multiple-threshold nonlinear ARDL estimator. Using the STIRPAT model [68], investigated the relationship between FD and EP in the. The results show that FD accelerated EP in the countries. The findings showed that energy had no impact on FD and EP.

In China, [66]- examined the relationship between FD and EP variables while accounting for energy usage and economic growth. According to the revelations, FD promoted EP throughout the nation, looked on the interactions between FD and EP in Argentina between 1971 and 2018. Estimates since the DOLS, ARDL, CCR, and FMOLS show that FD enhanced EP in the nation through lowering carbon emissions [68]. Looked on the connections between financialization and environmental impact in BEM economies between 1995 and 2016. The findings demonstrated that financialization has a negative impact on EP around the globe. Between [67] examined the link between FD-EP in 24 different nations.

RETRACTED

Since the detection, high emissions have caused EP to gradually decline [62, 69] had studied Pakistan from 1972 to 2018 by the year 2020. Because negative shocks in FD had the biggest impact on carbon spread, the review exhibited that there was a lopsided connection among FD and EP. From 1983 to 2019 [70], looked into the connection among FD and EP variable in Bangladesh. The results showed that FD did not have any significant ties to EP. From 1980 to 2019. The estimates of ARDL, FMOLS, DOLS, and CCR provided by the study suggested that EP in the nation was unaffected by FD. Between 1991 and 2015, the FD-EP connections of 58 nations were investigated. The findings indicated that bank-based FD improved the countries’ EP; Market-based FD and EP, on the other hand, did not share many similarities. Additionally, a nonlinear connection was established between FD and EP.

[71] said that their current study makes an effort to investigate the factors that affect CO_2_ emissions per person while taking into account spatial impacts for a panel of 21 North American nations. The findings support the presence of spatial dependence in carbon dioxide emissions per person and its underlying causes. All of the hypothesized factors were found to have negative environmental implications, although per capita income had a positive effect. Similarly, another study [72] the current study conducts regional analysis from 1990 to 2018 to examine the environmental impacts of trade, Renewable Energy Consumption (REC), and industry value-added in South America. The local CO_2_ emissions are positively impacted by per-capita income. It also negatively affects the environment in neighboring nations in terms of consumption-based CO_2_ emissions, but not in terms of territory-based CO_2_ emissions. Moreover, China is the nation that produces the most pollution overall, and the environmental Kuznets curve (EKC) theory has been extensively researched there. As a result, our goal is to analyses empirical research that tested the EKC hypothesis in China using various pollution proxies and region samples. Establishing an N- or an inverted U-shaped relationship between pollution and economic growth will support the EKC hypothesis [73]. Any nation’s ecology could benefit from the agriculture industry. The goal of this study is to examine the environmental Kuznets curve (EKC) theory’s validity while taking Saudi Arabia’s energy consumption and agricultural sector’s contribution to national GDP into account. The magnitudes of the effects of rising and falling agricultural GDP shares are statistically found to have differing effects on CO_2_ emissions, with rising agricultural GDP shares having a bigger impact than declining agricultural shares [74].

RETRACTED

EP benefited from the findings for FD; But there remained no obvious link among the group of nations. The top ten economies with the highest mineral resources from 1990 to 2019 were examined [75] which looked at these economies. With regard to environmental contamination, financial services were shown to reduce mineral resource rent. According to the study’s threshold findings, found that an increase in FD enhanced EP in the countries by reducing emissions. He came at this conclusion by studying the BRICS economies from the year 2000 to 2018. [6] investigated the interactions between FD and EP in the N-11 nations between 1990 to 2016. The study’s application of contemporary econometric techniques shown how EP in the nations suffered from FD. From 1990 to 2016. [72] investigated the economies of South Asia, the results of examination show that FD is detrimental to EP in the nations [75]. The discovery caused EP in the countries to worsen [55] investigated if FD in the Asia-Pacific area supported the EKC theory. The results confirmed the U-shaped connection among FD and EP in the area. Furthermore, it remained shown that FD and EP are related. [76] analyzed the FD-EP correlations of 83 economies Overall estimations indicate that EP was not considerably impacted by financial market developments. Moreover, there were differences across nations in the controlling and nonlinear impacts of financial arcade modifications regarding EP.

Another study [4] The purpose of this study is to determine how country risks and the utilization of renewable energy affect environmental quality. Data from 1990 to 2018 are used in this study, which looks at the MINT (Mexico, Indonesia, Nigeria, and Turkey) countries. Cross-sectional autoregressive distributed lag (CS-ARDL) is used as the main model, with common correlated effects mean group (CCEMG) and augmented mean group (AMG) being used for robustness checks. The empirical findings demonstrate that (i) urbanization, political risk, economic expansion, and trade openness all contribute to a rise in the ecological footprint; (ii) The use of renewable energy sources and economic and financial risks have a good impact on environmental quality; (iii) there is a one-way causal relationship between the environmental pollution and economic growth, financial risk, political risk, urbanization, and trade openness. Moreover, another side the [8]- again argue with another study that they use the Fourier approaches of stationarity, co-integration, causality along with the long-run estimators of fully modified and dynamic least squares to examine the environmental aspects of resource productivity, environmental-related technologies, and export intensity over the period of 1990–2021. The study is motivated by G-7 ambitious transition to circular economy through the reduction of consumable nonrenewable resources and carbon neutrality by 2035. It’s interesting to note that the results showed that, given the two long-run estimators, an increase in raw material productivity results in a drop in greenhouse gas emissions of between 61 and 70 percent Additionally, the Fourier Toda Yamamoto and causality approaches provide a strong inference coupled with an implication of the long-term outcomes for all the elements under consideration. In light of this insight, pertinent policy initiatives were identified to help Finland’s decision-makers further pursue the circular economy and the carbon zero aim.

RETRACTED

In the context of renewable energy, this study intends to examine the relationships between value orientation, utilitarian advantages, collectivism, the reason for adoption, attitude towards RE, and adoption intention. The study examines survey information from 359 Pakistani consumers who own solar-powered homes. To assess hypotheses, a method known as structural equation modelling is used. According to empirical results, value orientation has a positive and significant impact on both the motivation for adopting RE and one’s attitude towards RE. The utilitarian benefit similarly has a positive and significant impact on one’s attitude towards RE [77]. Furthermore, adoption of renewable energy is a difficult process that is affected by many different variables. Previous research hardly ever looked at Shandong province’s social acceptance of renewable energy from a Chinese standpoint. The public’s perception of renewable energy must be ascertained through thorough study in order to close this gap. By adding three new variables risk perception, environmental concern, and belief about the costs of renewable energy we expanded the theory of planned behavior [78].

This study tries to pinpoint the factors that influence consumers’ decisions to purchase environmentally friendly appliances for their homes. In the setting of an emerging economy, this study examines the relationships between environmental knowledge (EK), consumer attitude (CAT), green trust (GT), and purchase intention (PI). In this study, survey information from 331 Pakistani consumers who utilize energy-efficient household goods is analyzed. The formulated hypotheses are evaluated using SEM. Empirical results indicate that EK considerably and favorably affects CAT and green trust. Similar to CAT, PI is negatively and negligibly impacted by CAT. Green trust, on the other hand, is considerably and favorably associated to PIs. [77] again argue with three new variables environmental knowledge, environmental concern, and views about the advantages of solar energy were introduced to the study’s theory of planned behavior. A thorough questionnaire survey was used to gather primary data from 847 respondents in the Hebei Province. The data were examined using structural equation modelling. According to empirical findings, views about solar energy’s advantages, environmental awareness, subjective norms, perceived behavioral control, and attitude all have a favorable impact on consumers’ intentions to purchase solar energy. On the other hand, the intention to purchase solar energy was unaffected significantly by environmental concerns [79].

RETRACTED

The purpose of the current study is to assess how well Pakistan’s small-scale industry has developed since SHS was implemented. Purposive sampling was used to choose respondents for an all-encompassing questionnaire survey. We go one step further and examine the regulating function of technological knowledge and understanding between the adoption of SHS and the monetary implementation of small-scale enterprise. Using a sample of 357 respondents using the partial least square structural equation modelling (PLS-SEM) method, we validate the model. The findings show that low-cost energy supplied by SHSs improves Pakistan’s quality of energy supply and has a progressive and significant relationship with the development of small-scale manufacturing [80].

After all discussion in literature review we found our gap on environmental pollution is a difficult problem, future study must take a variety of environmental contamination proxies in growing countries into consideration. It is recommended that elements be taken into account as soon as data is available for the construction of the financial development (FD) and green investments (GI) directories. Finally, comparable study must to be carried out for other developed and developing countries.

## Martials and methods

Investment (GI) metrics are based on the use of renewable energy, technological advancements, and domestic credit provided by banks to the private sector is represented by financial Development (FD) and domestic credit to private sector; EG is measured by per capita GDP [81] The CO_2,_ environmental pollution (EP) is measured in kilo tons (kt). The study covered the time G-7 from 1997 to 2021.

RETRACTED

The description of the variable, the measuring unit, and the data source are depicted in Table 1. In this section, we discuss the nonlinear autoregressive distributed lag (NARDL) model of [82] are discussed in relation to asymmetrical causality. The asymmetric effect of the variables on carbon emissions is examined using the nonlinear ARDL method. Listed below are the goals of this evaluation method: i) Nonlinear asymmetry and conintegration are two concepts that can be combined into one Equation.

**Table 1:** Variables description.

Variable	Unit of Measurement	Sources
**Environmental Pollution (EP)**	Metric tons per capita	World Bank
**1-Economic Growth**	Per capita GDP	World Bank
**2-Green Investment (GI)**		
a)-Technological innovations	No. of patent for non-resident and resident computed by PCA	World Bank
b)- consumption of Renewable energy	(% of total final energy consumption)	World Bank
**3-Financial Development (FD)**		
a)-Domestic credit to private sector by banks	Percentage of GDP contain by PCA	World Bank
b)-Domestic credit to private sector	Percentage of GDP contain by PCA	World Bank

When the decomposed variables exhibit positive and negative variations, the NARDL model examines the positive and negative effects on the dependent variable. ii) The model performs well with small sample sizes. The fact that the variables do not have to be added in the same order makes it adaptable.

### Environment pollution

Pollution in the environment referring to [83] the fundamental data on CO_2_ (carbon dioxide emissions) were used to create a comprehensive environmental pollution.

### Green investment (GI)

By expanding technological innovation capabilities, upgrading the industrial structure, and improving the efficiency of energy conservation and emission reduction, green investment can reduce environmental pollution. The environmental crisis is the result of the environmental deterioration caused by a variety of forms of pollution, the rapid exploitation/utilization of natural resources.

### Technology innovations

The economic process by which new technologies are incorporated into production and consumption is known as technological innovation. According to [84], green innovations have the potential to effectively reduce environmental pollution as well as the negative effects of processes that use resources (and energy) and create sustainable development. Even though innovation is a well-defined concept, it has many different meanings for many people, especially in the academic and business communities. I use technological innovations, such as patent applications from residents and nonresidents, as a proxy for green investment.

RETRACTED

### Renewable energy consumption

Energy that comes from natural sources and is replenished at a faster rate than it is used is called renewable energy. Types of generated energy from the sun. Wind power. Hydro power. Tidal power.

### Financial development

In order to facilitate EP expansion, FD encourages investments in environmentally friendly technology. A robust financial sector encourages sustainability and energy efficiency by supporting the development of residential products that use less energy [65].

### Methods

The Schwarz criterion, which was proposed by [85] and stipulates that the maximum number of breaks points should be 2, has been applied to the breaks points assurance.

$$EP=\beta 0+\beta 1\;{GI}_{it}+\beta 2{GDP}_{it}+\beta 3\;{FD}_{it}+\mu_{it}$$ (1)

Where EP, GI, FD, and EG represent, respectively, environmental pollution, green investment, economic growth and (FD) financial development. We assert that these variables are major contributors to clean environmental pollution and key production factors.

#### Cross sectional dependence (CD)

The issue of cross-sectional dependence has recently come up in econometrics analysis because of spillover effects like shock, undetected components, and spatial dependency that might affect long-term policy consequences by spitting over dependent on a particular state [86] Because of this, the outcomes without a CD test may be skewed and unpredictable [87]. We initially check the data for CD using the previously mentioned concern reasons [83]. The alternative explains the existence of cross-sectional dependency and vice versa.

#### Unit root tests

We performed a variety of panel unit tests to verify the stationarity condition of the variables. In our analysis on the designated panel data, they include the (CIPS) test [88]. The "first-generation unit root" cannot report the cross sectional dependence issues, so we used second-generation unit tests. If the variables are unified in the same order in both tests, the null hypothesis can be rejected.

Eq (2) show change in logarithmic and positive and negative changes too in descriptive variables will be written as:

$$InEP_{it}=a_{it}+\delta_{t}\;InEP_{it-1}+\beta^{+}InGI_{it}^{+}+\beta^{-}InGI_{it}^{-}+\beta^{+}InFD_{it}^{+}+\beta^{-}InFD_{it}^{-}+\beta^{+}InEG_{it}^{+}+\beta^{-}InEG_{it}^{-}u_{it}$$ (2)

Where u is the error term with time t, u is the intercept, s are the variable coefficients, ln is the natural logarithm, and is the trend effects. The framework of EP. (4)’s nonlinear autoregressive distributed lag (NARDL) may be stated as:

$$\Delta InEP_{it}=\mu +\delta_{t}InEP_{it-1}+\theta^{+}InGI_{it-1}^{+}+\theta^{-}InGI_{1-it}^{-}+\vartheta^{+}In{FD}_{1-it}^{+}+\vartheta^{-}In{FD}_{1-it}^{-}+\omega^{+}InEG_{1-it}^{+}\omega^{-}InEG_{1-it}^{-}+$$ (3)

$$\sum_{j=1}^{z}+\alpha_{j}\Delta InEP_{it-j}+\sum_{j=0}^{z}(\pi_{j}^{+}+\Delta InGI_{it-j}^{+}+\pi_{j}^{-}\Delta InGI_{it-j}^{-})+$$

$$\sum_{j=0}^{z}(\vartheta^{+}In{FD}_{it-1}^{+}+\vartheta^{-}In{FD}_{it-1}^{-})$$

$$+\sum_{j=0}^{z}(\omega^{+}InEG_{it-1}^{+}\omega^{-}InEG_{it-1}^{-}+\epsilon_{it}$$

The continuity Equation may be used to predict the short-run NARDL elasticities using error correcting mechanism:

$$\Delta InEP_{it}=\mu +\sum_{j=1}^{z}+\alpha_{j}\Delta InEP_{2it-j}+\sum_{j=0}^{z}(\pi_{j}^{+}\Delta InGI_{it-j}^{+}+\pi_{j}^{-}\Delta InGI_{it-j}^{-})$$ (4)

$$\sum_{j=0}^{z}(\vartheta^{+}In{FD}_{it-1}^{+}+\vartheta^{-}In{FD}_{it-1}^{-})+\sum_{j=0}^{z}(\omega^{+}InEG_{it-1}^{+}+\omega^{-}InEG_{it-1}^{-})+$$

$$+ØECM_{it-1}{+\epsilon }_{it}$$

The effect of variables GI, FD, and EG can be putrefied into 2 parts, positive and negative

$$InGI_{it}=InGI_{0}+In{GI}_{it}^{+}+In{GI}_{it}^{-}$$ (5)

$$InFD_{it}=InFD_{0}+InFD_{it}^{+}+InFD_{it}^{-}$$ (6)

$$InEG_{it}=InEG_{0}+InEG_{it}^{+}+InEG_{it}^{-}$$ (7)

Where ***InGI***_**0,**_ ***InFD***_**0**_, and ***InEG***_**0**_ represent the random initial value and $In{GI}_{it}^{+}+In{GI}_{it}^{-},InFD_{it}^{+}+InFD_{it}^{-}$ and $InEG_{it}^{+}+InEG_{it}^{-}$ indicate systems that compute fractional sums of positive and negative^-tv^ variations, correspondingly, and are characterized as

$$InGI_{j}^{+}=\sum_{j=1}^{t}\Delta In{GI}_{it}^{+}=\sum_{j=1}^{t}max(\Delta InGI_{j,}\;0),$$

$$InGI_{j}^{-}=\sum_{j=1}^{t}\Delta In{GI}_{it}^{-}=\sum_{j=1}^{t}min(\Delta InGI_{j,}\;0){+\epsilon }_{t}$$ (8)

$$In{FD}_{j}^{+}=\sum_{j=1}^{t}\Delta In{FD}_{it}^{+}=\sum_{j=1}^{t}max(\Delta In{FD}_{j,}\;0),$$

$$In{FD}_{j}^{-}=\sum_{j=1}^{t}\Delta In{FD}_{it}^{-}=\sum_{j=1}^{t}min(\Delta In{FD}_{j,}\;0){+\epsilon }_{t}$$ (9)

$$InEG_{j}^{+}=\sum_{j=1}^{t}\Delta InEG_{it}^{+}=\sum_{j=1}^{t}max(\Delta InEG_{j,}\;0),$$

$$InEG_{j}^{-}=\sum_{j=1}^{t}\Delta InEG_{it}^{-}=\sum_{j=1}^{t}min(\Delta InEG_{j,}\;0){+\epsilon }_{it}$$ (10)

The implications of the asymmetric cumulative dynamic multipliers on *InEP*_*t*_ of a unit change $In{GI}_{t}^{+},In{GI}_{t}^{-}t$, $InFD_{t}^{+}+InFD_{t}^{-}$ and $InEG_{t}^{+}+InEG_{t}^{-}$, can be obtained, respectively, as follows:

$$m_{h}^{+}=\sum_{j=0}^{h}\frac{\delta InEP_{2t+j}}{\delta In{GI}_{it-1}^{+}},m_{h}^{-}=\sum_{j=0}^{h}\frac{\delta InEP_{2t+j}}{\delta In{GI}_{it-1}^{-}}$$

$$m_{h}^{+}=\sum_{j=0}^{h}\frac{\delta InEP_{2t+j}}{\delta In{FD}_{it-1}^{+}},\;m_{h}^{-}=\sum_{j=0}^{h}\frac{\delta InEP_{2t+j}}{\delta In{FD}_{it-1}^{-}},$$

$$m_{h}^{+}=\sum_{j=0}^{h}\frac{\delta InEP_{2t+j}}{\delta In{EG}_{it-1}^{+}},\;m_{h}^{-}=\sum_{j=0}^{h}\frac{\delta InEP_{2t+j}}{\delta In{EG}_{it-1}^{-}}h$$ (11)

Note: as *h* → ∞, then $m_{h}^{+}$ →*β*^+^ and $m_{h}^{-}$ →*β*^−^, where *β*^+^ and *β*^−^, are calculated as β+=−θ−ρandβ−=−θ−ρ, respectively.

RETRACTED

#### Principal component analysis

To construct PCA, we have referred to the studies of [51, 89] In this work, we do PCA (Principal Component Analysis) of all the proxies of green investment using annual data on consumption of renewable energy and technology advancement.

In PCA, the kth feature indices are stated as:

$$GI_{k}=M_{k1}N_{1}+M_{k2}N_{2}$$ (12)

GIk stands for green investment in this case. Mk and Nk, respectively, stand for the parameters’ respective weights. The values of green investments (consumption of renewable energy and technological advancement) are indicated by the numbers N_1_, N_2_, etc.

Additionally, we use domestic bank credit to the private sector and domestic credit to the private sector (two proxies for financial development) and do PCA on this data before naming it financial development (FD) by designing the study.

Using the PCA method, we created the following financial development (FD) index equation:

$$FD_{h}=O_{h1}P_{1}+O_{h2}P_{2}$$ (13)

FDh stands for the financial development index in this context. Oh1 and P1h, respectively, stand for the parameters’ respective weights. The values of the financial development indicators are indicated by P_1_, and P_1_,

## Results and discussion

This research sought to examine the relationship between GI, EG, FD, and EP both theoretically and empirically. Different econometric methods were used to analyses the data set of the G-7 economies. In addition to doing CD tests, panel unit root tests, and various co-integration tests, we also used NARDL to test long- and short-term relationships.

Table 2 presents the results of the CD check. The results showed that CD exists in our data set and the alternative hypothesis was accepted at 1% significance.

**Table 2:** Cross sectional dependence test.

Variables	CD-Test	P-value
EP	10.22	0.000***
GI	14.54	0.000***
FD	11.77	0.000***
EG	15.23	0.000***

Note

***, **, * indicate significance at the 1%, 5%, and 10% levels, respectively

We employ second-generation unit root tests, like CIPS tests, to verify the stationary state in our data since we have proven the existence of CD in it. Table 3 presents the results of the tests stated above. According to the results of the CIPS unit root test, all variables are stationary at the initial difference. The findings of CD test and 2^nd^ generation unit root test are consistent with the findings of [51, 90].

RETRACTED

**Table 3:** Panel unit root analysis.

Variables	CIPS	
	At level	First difference
EP	0.876	3.432
GI	2.332	2.884
FD	-1.246	3.214
EG	-1.874	4.321

### Panel cointegration analysis

Table 4 shows that to ascertain if the dependent and independent variables have a long-term relationship, we utilized the most prominent panel co-integration tests, namely the Pedroni and Kao [91, 92]. In every instance, we apply individual intercept, followed by weighted statistics test, statistics test, and Schwarz Info criterion, and we also employ lag length from the Swiss info criterion.

**Table 4:** Pedroni (Engle-Granger based) test.

**ALTERNATIVE HYPOTHESIS: COMMON AR COEFS. (PANEL A: WITHIN-DIMENSION)**					
Panel co-integration test		Individual intercept			
		Prob.	Weighted Statistics		Prob.
Panel v-Statistic		0.145	0.702		0.241
Panel rho- Statistic		0.698	0.623		0.733
Panel PP- Statistic		0.055*	-1.766		0.038*
Panel ADF- Statistics		0.008*	-2.260		0.011*
**ALTERNATIVE HYPOTHESIS: INDIVIDUAL AR COEFS. (PANEL B: BETWEEN-DIMENSION)**					
Panel co-integration test	Individual intercept				
	Prob.			Statistics	
Panel rho- Statistic	0.966			1.833	
Panel PP- Statistic	0.027*			-1.926	
Panel ADF- Statistics	0.015*			-2.156	

Basis: Calculation by authors. The lag length was selected by the Schwarz Info criterion.

Note

***, **, * indicate significance at the 1%, 5%, and 10% levels, respectively

Two-dimension test statistics between and within dimension test statistics are reported by the Pedroni panel co-integration test analysis. Panel co-integration’s H_0_ and H_1_ were contrasted. The Pedroni panel co-integration tests’ findings indicate that the H_0_ of no co-integration can be ruled out at a level of significance of 10%, 5%, or 1%. The findings of panel co-integration are consistent with the findings of [4, 43].

Table 5 displays the results of the probability-based Augmented Dickey-Fuller (ADF) Kao panel co-integration test, which was also performed; it produces a significant result of 0.089, which is followed by residual variance and HAC variance. All relevant variables are assumed to have a long-term relationship based on the findings of co-integration analysis. The Kao panel co-integration test results suggest that the null hypothesis of no co-integration may be rejected at the 10%, 5%, or 1% level of significance. There is a long-term association between environmental pollution in G-7 countries, green investment, financial development, and GDP, as predicted by Table 5.

**Table 5:** Kao (Engle-Granger-based) test.

ADF (Prob.)	Residual variance	HAC variance
0.039*	0.084	0.089

Source: Calculation by authors. The lag length was selected by Modified Hannan-Quinn

Note

***, **, * indicate significance at the 1%, 5%, and 10% levels, respectively

RETRACTED

### Panel NARDL long run and short run estimation

Table 6 displays the outcomes of the NARDL model’s long-run and short-run estimations. The essential goal of the review is to affirm the nonlinear imbalance connection between green venture, ecological contamination, CO_2_ discharges, Gross domestic product, and monetary turn of events. The calculated coefficients of the positive and negative sums for the increment and decrease of the decomposed variables are depicted in the long-term model’s output. The cointegration test confirmed the imbalance between the decomposed variables and CO_2_ emissions over time. Long-term NARDL data serve as the foundation for green investment coefficient estimations with positive and negative shock.

**Table 6:** Long run and short run estimation NARDL.

Variable	Coefficient	Std. Error	t- statistics	Prob
FD_POS	0.6108	0.0883	6.9143	0.000
FD_NEG	-0.0734	0.0544	-1.4199	0.1590
EG_POS	0. 4582	0. 1531	2.9978	0.0448
EG_NEG	0. 4739	0.0612	0.7471	0.0000
GI_POS	0.3804	0.1688	2.2859	0.0573
GI_NEG	0.6872	0.1685	5.1546	0.0000
**Short Run**				
ECT	-0.4672	0.2006	-2.5572	0.0228
d(EP(-1))	0.0545	0.1501	0.3635	0.7170
d(FD_POS)	0.1320	0.0264	4.9924	0.0424
d(FD_NEG)	0.5035	0.1768	2.8360	0.0584
d(EG_POS)	0.2552	0.1045	2.4846	0.0541
d(EG_NEG)	0.2513	0.1221	2.0576	0.0425
d(GI_POS)	0.1436	0.0398	4.2307	0.0063
d(GI_NEG)	-0.1365	0.0246	-5.5481	0.0007

According to the long-run results, the estimates for Green Investment (GI) increases and reductions are both positive and negative. According to the findings, a one-unit increase in green investment (GI-POS) also produces a 0.3804 increase in CO_2_ emissions, whereas a one-unit negative shock in green investment (GI-NEG) leads in a 0.6872increase in CO_2_ emissions in the long run. Additionally, we discover that improvements in green investments (GI-POS) have a greater effect on CO_2_ emissions than detriments (GI NEG). These studies are aligned with [16, 21, 39, 93, 94].

Our findings provide more evidence for the long-term asymmetry between financial development and environmental performance. According to the findings, a one-unit increase in financial development (FD-POS) causes a 0.6108 decrease in CO_2_ emissions, whereas a one-unit fall in financial development (FD-NEG) causes a -0.0734 decrease. Thes findings are aligned with the previous studies of [95–98]. The finding confirmed that FD-POS has a bigger influence on environmental performance when compared to FD-NEG. Moreover, FD also supports spending on R&D projects that remain connected toward (EP) environmental pollution.

RETRACTED

Similar conclusions are found for economic growth expansion and environmental performance, where we uncover an uneven relationship between the two. It has been determined that a one-unit rise in GDP growth (EG-POS) results in an increase in environmental pollution (CO_2_ emissions) of 0. 4582, whereas a one-unit drop in EG growth results 0. 4739 in a decrease in environmental pollution (CO_2_ emissions). The results are aligned with [99–101]. Positive shocks of EG are less harmful to the environment than negative ones. However, the correlation between EG and environmental pollution shows that a decline in EG has a higher effect on pollution than a rise in economic development, FD is 0.3804.

Findings demonstrate (Table 6) a short-term inverse link between environmental pollution (EP), economic growth, and green investment. In short run analysis, it is found that we strongly need clear and comprehensive policy to reduce environmental pollution and increase green investment to improve environmental pollution with EG is 0.1436 and financial development is 0.1320.

According to the findings, a one-unit increase in green investment (GI-POS) also produces a 0.1436 increase in CO_2_ emissions (EP), whereas a one-unit negative shock in green investment (GI-NEG) leads in a -0.1365 increase in CO_2_ emissions in the short run. Additionally, we discover that improvements in green investments (GI-POS) have a greater effect on CO_2_ emissions than detriments (GI NEG). However, if green investment has negative shocks, it can be difficult to control environmental performance. Since it is difficult to provide accurate estimates for calculations without them, long-term barriers result, empirical data show that government should make sensible judgements and regulate all elements in the short term. Our findings provide more evidence for the long-term asymmetry between financial development and environmental performance. According to the findings, a one-unit increase in financial development (FD-POS) causes 0.1320 a decrease in CO_2_ emissions, whereas a one-unit fall in financial development (FD-NEG) causes a 0.5035 decrease. The fact that environmental pollution reduces CO_2_ emissions shows that it is challenging to regulate all the variables influencing environmental pollution activities in the G-7 nations. It has been determined that a one-unit rise in GDP growth (EG-POS) results in an increase in environmental pollution (CO_2_ emissions) of 0.2552, whereas a one-unit drop in EG growth results 0.2513 in a decrease in environmental pollution (CO_2_ emissions). Positive change of EG is less harmful to the environment than negative ones. However, the correlation between EG growth and environmental pollution shows that a decline in EG growth has a higher effect on pollution than a rise in economic development.

RETRACTED

The dynamic multiplier of environmental pollution, EP (Fig 1) demonstrated the short-run and long-run impact of positive and negative shocks of green investment (GI), financial development (FD), and economic growth (EG) on environmental pollution (EP). The dim dotted line represents the cumulative dynamics of explanatory variables, financial development, green investment, and economic growth with respect to an increase (positive shock) in explanatory variables while the dark dotted line denotes the effect of negative shocks of explanatory variables on environmental pollution. The thick line between the 95 percent confidence intervals gives the difference between positive and negative responses. The overall impression is that response of environmental pollution to positive and negative shocks of GI, EG, and FD are detected with a rapid reaction for first year. Whereas the reaction to the positive and negative shocks is absorbed after approximately 2 years to reach an equilibrium state. Moreover, an overall positive relation between variables because positive change in FD, GI, and EG have dominating positive effects on EP.

**Fig 1:** Environmental pollution (EP) dynamic multipliers. Dim line—-Positive change, Dark line——Negative change, Thick line——asymmetry.

## Conclusion and policy implication

The core purpose of the study to analyze the asymmetric effect of green investment, financial development and economic growth on environmental pollution in G-7 countries. Applying Panel NARDL, the finding affirms that the positive change of green investment (GI) has a significant and positive influence of environmental pollution. While the negative change of green investment has a positive and significant relationship with environmental pollution in G-7 countries. However, the positive shock of financial development (FD-POS) is positive association with environmental pollution in the long-run, while negative change in financial development has negative impact with environmental pollution.

More ever, in Fig 2 shows that the positive and negative change pf economic growth EG-POS) have positive and significant effect on environmental pollution in the long run.

**Fig 2:** Graphical presentation of results findings.

G-7 countries, including the United States, the United Kingdom, Canada, Japan, France, Italy, and Germany, have serious environmental problems. To control these problems, we have used different econometric techniques to overcome these issues. According to the results of the asymmetric analysis, the NARDL estimator’s relationship was used to investigate the elastic properties of the response variable. Green investments increased environmental pollution in G-7 nations, which had both a long-term and short-term effect on carbon dioxide mitigations. In addition, environmental pollution has decreased in G7 nations as a result of its positive effect on carbon dioxide emissions, which is measured by the proxies of private sector banks and public sector banks. Similarly, in both the long and short term, energy efficiency contributed to environmental pollution. For the G7, the relationship between revenue and (EP) environmental pollution remained subsequently show N-shaped establishment. Green investments were linked to environmental degradation in the causal directions among the variables.

RETRACTED

However, we also confirm that environmental pollution and financial growth were discovered. To help raise the nation’s declining rate of clean energy consumption, it should be suggested that energy from renewable sources be included in its various energy mixes. In addition, increasing investments in technological advancements is an efficient strategy that has the potential to encourage environmental pollution in the G-7. Additionally, increasing investments in emission-reduction research and development could reduce pollution in the country.

Additionally, the financial sector’s developments demonstrated the significant impact on environmental pollution. Countries with this impact on financial development have lower levels of environmental pollution. Conforming to [6] the research commends that industries that incorporate environmental pollution into their accomplishments receive credits. In order to limit the negative effects of financial sector development on environmental pollution, it is also crucial that consumers are encouraged to use less carbon-intensive household goods. In addition, the nation’s public sector financial institutions ought to improve their financing of investments in the development of energy-efficient technologies and products, as well as research and development pertaining to the transition to clean energy and energy expansion through green investment. Furthermore, giving customers finance would encourage the use of fuel domestic appliances, which would result in an increase in environmental pollution in G-7 countries. According to [64] well-established finance systems can raise private sector spending on the study and creation of less carbon-intensive technologies in 2021. They can also help identify and remove obstacles that affect user behavior and firms’ early aspirations for sustainable energy.

RETRACTED

For the G-7 to benefit from the benefits associated, they should concentrate on improving their financial systems. Also, the links show how environmental degradation and energy use are positively related. It makes sense for the nation to convert to utilizing energy from clean, well-established environmentally favorable sources because it is largely dependent on energy from filthy sources. Using clean energy is advantageous for countries since it would reduce their dependency on unreliable energy sources and help the G-7 countries reduce environmental damage. In addition, the G-7 nations ought to make an effort to direct their aid toward the clean energy sector. It is represented by financial investment, technical expertise, or green energy technologies, all of which are intended to reduce (EP) environmental pollution in nations. In addition, the G-7 nations ought to relax their green investment policies in order to raise the quality of inputs that can support the production of clean energy. As a result, the transactions may reduce environmental pollution and be environmentally friendly.

Finally, this shows that raising green investment may affect the nation’s environmental pollution in both favorable and unfavorable ways. To achieve this, the country should encourage ecologically friendly manufacturing and consumption practices. Also, if it implements industrial methods that utilize less carbon, the nation may turn into a net exporter of clean products and services. The institutional frameworks required to enhance mutually environmental pollution and (EG) economic growth must be built because G-7 economy is still in its infancy. One of the study’s shortcomings was the absence of data. This limitation limited the study’s coverage to the period from 1997 to 2021.

The collected results give us the chance to offer some worthwhile policy suggestions to the G7 nations. Firstly, the government needs to put laws into place that encourage green investment by funding energy-saving technology research, development (for businesses), and adoption (by businesses and families). The transition from high to low energy demanding facilities nevertheless necessitates enormous costs, which strain the budget of economic agents even though the G7 countries are categorized as high-income groups. Therefore, policymakers should establish a reasonable cost-sharing plan between the government and economic actors. Secondly, financial development combined with green investment can be a powerful strategy for reducing carbon dioxide emissions. The G7 nations have a long history of being heavily dependent on green investment sources, despite recent increases in the shares of green investment in both production and consumption. In order to improve incentives for producing enterprises, governments should create favorable feed-in tariff structures and offer additional tax breaks. Environmental awareness-raising initiatives (for homes) should be developed with regard to consumers. Furthermore, the government should also keep enforcing strict environmental laws and take steps to safeguard the environment while knowledge is being developed. Better environmental quality could be attained by promoting the use of cleaner, more effective production methods and energy sources.

RETRACTED

This restriction led to the review being limited to the years 1997–2021. Due to data constraints, the researchers were unable to calculate the financial development and green investments indices using all of the needed criteria. Future research must include a range of environmental contamination proxies in emerging countries meanwhile environmental pollution is a complex issue. It is advised that aspects be incorporated into the computation of green investments (GI) and financial development (FD) directories as quickly as data is available. Lastly, additional research on other developing nations should be carried out in order to assist in examining the results’ heterogeneity.

Abbreviations Explanation Symbols Explanation

## Abbreviations

EP: Environmental Pollution, Carbon dioxide emissions
EG: Economic growth
FD: Financial development
PCA: Principle component analysis
CD: Cross sectional dependence
GHG: Greenhouse gas emissions
NARDL: Nonlinear autoregressive distributed lags
FMOLS: Fully modified ordinary least square
GW: Gigawatt
GI: Green investment
kt: Kiloton
